# Compound W-Net with Fully Accumulative Residual Connections for Liver Segmentation Using CT Images

**DOI:** 10.1155/2022/8501828

**Published:** 2022-02-09

**Authors:** Mahmoud Abdelazim Khattab, Iman Yi Liao, Ean Hin Ooi, Siang Yew Chong

**Affiliations:** ^1^School of Computer Science, University of Nottingham, Semenyih 43500, Malaysia; ^2^School of Engineering, Monash University, Sunway, 47500, Malaysia

## Abstract

Computed tomography (CT) is a common modality for liver diagnosis, treatment, and follow-up process. Providing accurate liver segmentation using CT images is a crucial step towards those tasks. In this paper, we propose a stacked 2-U-Nets model with three different types of skip connections. The proposed connections work to recover the loss of high-level features on the convolutional path of the first U-Net due to the pooling and the loss of low-level features during the upsampling path of the first U-Net. The skip connections concatenate all the features that are generated at the same level from the previous paths to the inputs of the convolutional layers in both paths of the second U-Net in a densely connected manner. We implement two versions of the model with different number of filters at each level of each U-Net by maximising the Dice similarity between the predicted liver region and that of the ground truth. The proposed models were trained with 3Dircadb public dataset that were released for Sliver and 3D liver and tumour segmentation challenges during MICCAI 2007-2008 challenge. The experimental results show that the proposed model outperformed the original U-Net and 2-U-Nets variants, and is comparable to the state-of-the-art mU-Net, DC U-Net, and Cascaded UNET.

## 1. Introduction

The liver is the largest substantive organ of human body. It maintains important life activities such as detoxification and metabolism. Computed tomography (CT) is a common modality to detect liver and liver lesions. Liver segmentation is important for the formulation of treatment plan and for the evaluation of the follow-up treatment effect. As the manual segmentation is error-prone and time-consuming, automatic liver segmentation methods have been extensively studied [1–3].

Liver segmentation is still a challenging task, due to the variability of organ's shape and size and similar intensity values among neighbouring organs and tissues, such as the heart, the stomach, the kidneys, and the abdominal wall. On the other hand, a liver has a crucial role in metabolic processes; therefore, it is essential to perform a fast and accurate diagnosis in case of any disease. Moreover, with the improvement of different medical imaging techniques, the focus is placed on the application of noninvasive diagnostic methods, before performing a painful, invasive examination (e.g., biopsy). Out of different liver pathologies, liver cancer is the fifth most commonly occurring cancer in 2018 world-wide, according to the World Health Organisation and others [4–7]. Therefore, a continuous effort is required to develop efficient and automatic segmentation methods, which may support the diagnostic process and facilitate the treatment decision-making.

Liver segmentation task has been introduced as a challenge for many conferences, e.g., MICCAI 2007, MICCAI 2008, and ISBI 2017. During these challenges, 3Dircadb1 and LiTS datasets were introduced for training and evaluation of the proposed approaches. The existing automatic liver segmentation methods are divided into two categories: pixel- or image-based segmentation and learning-based segmentation. Thresholding, region growing, edge detection, and graph cut [8–10] are some of the commonly used image-based segmentation methods, which directly segment images by the grey level, texture, and gradient. Most of them have low robustness, are prone to under or over segmentation, and are sensitive to initial seed selection; therefore, a sophisticated preprocessing is required. Therefore, in recent years, these methods are rarely applied to liver segmentation alone, but are usually used as a postprocessing for other methods.

The learning-based segmentation methods include statistical models, traditional machine learning methods, and deep learning methods. Supervised learning methods with pixel-wise binary classification usually performs better than the image-based segmentation methods, e.g., statistical models [11], active shape models (ASM), active appearance models (AAM) [9], level set-based methods [12], and atlas-based segmentation [13]. However, traditional machine learning methods, e.g., support vector machines (SVM) [14], and Adaboost [15], rely on extracting handcrafted image features, which is not efficient and subject to human bias. In contrast, deep learning methods extract image features automatically based on large training dataset without introducing human bias.

Convolutional neural networks have become the state-of-the-art in many fields especially for medical image analysis. U-Net was introduced in 2015 for the segmentation of neuronal structures in electron microscopic stacks. It works with binary crossentropy as a loss function for pixel wise classification, and the energy function is computed by a pixel-wise soft-max over the final feature map combined with the crossentropy loss function [16]. 2-bridged U-Net were proposed for prostate segmentation [17]. CNNs and deep learning approaches are widely used for liver segmentation and require significant number of training samples and preannotated masks as ground truth.

Segmentation processes are usually affected by the edge of the object. Although the skip connections in the conventional U-Net have effectively handled edge information to a certain extent, there are still room for improvement with the U-Net [18]. Firstly, the U-Net architecture duplicates low-resolution information of features. After pooling (i.e., downsampling), low-resolution information of features passes on to the convolution layer in the next stage. However, this low-resolution information of features is transferred by the skip connection of the U-Net as well. Duplication of low resolution information may then cause smoothing of the object boundary information in the network, which is more critical in the case of fuzzy object boundaries [19]. Another drawback of the U-Net architecture is that it may not sufficiently estimate high level features for high-resolution edge information of the input object. The U-Net use the skip connection to transfer high-resolution information; however, high resolution edge information does not pass through any convolution layers during transfer by the skip connection. Thus, higher level feature maps learned by the network do not contain enough information of the high-resolution edges of the input object. Consequently, in the conventional U-Net, high-level features are extracted disproportionately from low-resolution information [17, 20].

Many new models based on U-Net have been introduced to overcome the drawbacks of the original U-Net [16]. Stacked U-Net [21], V-Net [22], and bridged 2U-Net [23] are examples of the variants of the U-Net. Zhang and Xu [24] added a separated path to extract the global features and local features separately by reducing the number of convolutional channels of the contraction and expansion paths. It has led to a faster training process and improved the efficiency of the convolution kernel feature extraction [24]. Whilst the adjacent network with less number of parameters sped up the training process, it has a limited accuracy [25]. U-Net has also been integrated with other traditional registration and segmentation techniques such as conditional random field (CRF) to segment the liver tumour with limited number of samples [26, 27]. Christ et al. [28] proposed a cascaded CNN in 2D with a 3D dense CRF as a postprocessing step, to achieve higher segmentation accuracy whilst preserving low computational cost and memory consumption. Albishri et al. [29] cascaded 2 U-Net, one for the liver and one for tumour segmentation, with preprocessing Hounsfield units (HU) and Contrast Limited Adaptive Histogram Equalization (CLAHE). Liu et al. [30] proposed CR-U-Net, where the cascade U-Net is combined with residual mapping, and the second-level of cascade network is deeper than the first-level to extract more detailed image features and adopted morphological algorithms as an intermediate-processing step to improve the segmentation accuracy. Lu et al. [31] combined a 3D CNN with a Graph Cut (GC) algorithm for liver segmentation. Wang et al. [32] transformed the Dicom image format to Hounsfield Unit, then used a window of the specific HU for the liver before training with CNNs. They replaced the convolutional layers at each level with dense connection blocks where each dense block contains 5 U-Nets of 2 levels. Zhou et al. [33] combined U-Nets of varying depths into one ensemble architecture where different U-Nets share the same encoder but have separate decoders to encourage knowledge sharing. However, such architecture still suffers from two drawbacks. Firstly, the decoders are disconnected, and deeper U-Nets do not offer a supervision signal to the decoders of the shallower U-Nets in the ensemble. Secondly, the common design of skip connections used in the U-Net is unnecessarily restrictive, requiring the network to combine the decoder feature maps with only the same-scale feature maps from the encoder. While striking as a natural design, there is no guarantee that the same-scale feature maps are the best match for the feature fusion.

Recently, residual mapping has been used in combination with image segmentation architectures, which is an effective way to prevent overfitting and meanwhile to improve accuracy. Milletari et al. [22] combine residual learning with U-Net to construct V-Net for 3D image segmentation. Bi et al. [34] proposed a cascaded deep residual networks (ResNet) approach to segment the liver and liver lesions. As preprocessing, it converts the images to HU and applies data augmentation strategies including random scaling, crops, and flips and used 3D CRF and multiscale fusion for postprocessing. The network is pretrained firstly on the ImageNet dataset for parameter fine-tuning and is further fine-tuned with the liver dataset. On the other hand, Xu et al. [35] used HU as preprocessing and postprocessing 2D CRF and 3D CRF. ResU-Net added residual connections to each skip connection of the basic U-Net structure. Liu et al. [36] added attention block and residual block to the decoder path of the U-Net with adaptive dice loss function. It has helped increase the dice coefficient loss on LiTS dataset from 0.8365 to 0.9692 with all the residual and attention blocks. Seo et al. [20] included the residual path and a design of object-dependent upsampling to U-Net structure. The network avoids duplication of low-resolution information, estimates higher level feature maps that better represent high-resolution edge information of larger object inputs, and learns to extract even higher level global features for small object inputs. The testing accuracy on 3Dircadb dataset is 96.01 ± 1.8%, marking a relatively superior performance compared to other state-of-the-art.

The previously reviewed models can be categorized to three categories based on the number of U-Nets and the type of connections between the U-Nets. The first category contains the models based on one U-Net, e.g., mUNet [20] introduced a decovolutional block before the skip connection; [24] proposed an extra path for global feature extraction; residual U-Net [35] added residual connection between each two consecutive layers; densely connected U-Net [32] replaced the conv layer at each level to of the contraction path with dens block; [36] added attention module to each level of the expansion path. The second category contains the models that used 2 cascaded U-Nets, e.g., [28, 29] consist of two separated U-Net one for liver and one for tumor segmentation, whereas [34] adds CRF as a postprocessing technique. The third category contains the models that implemented 2 stacked U-Nets, e.g., [21] introduced 2 stacked U-Nets with N cut loss function; CRUNet [30] introduced 2 U-Nets with different depth and a morphological technique as intermediate process between the two; and [23] proposed one skip connection as a bridge between the 2 U-Nets.

In comparison, we propose a 2 stacked U-Net model. The model is not computationally expensive as it contains smaller number of layers compared to the Dense U-Net [32, 33] and less number of residual connections compared to [35]. The proposed model introduces 3 types of skip connections between the two U-Net in addition to the normal skip connection in each U-Net, whilst the bridge U-Net [23] used one bridge connection between the 2 U-Nets and [21, 30] contains only the skip connections of the original U-Net.

## 2. Materials and Methods

### 2.1. Data

3Dircadb1 (3D Image Reconstruction for Comparison of Algorithm Database) is created by Hôpitaux Universitaires France as a public dataset for researchers in medical image segmentation. The dataset is composed of 3D CT-scans for 20 patients with hepatic tumours in 75% of cases. For each patient, there are number of CT scans in addition to manually annotated mask for several structures of interests, e.g., liver, left kidney, right kidney, and hepatic tumours performed by clinical experts. All CT scans and masks are in DICOM format with pixel size (512 × 512). The total numbers of CT scans are 2823. We adopted two augmentation techniques as in [37] to increase the number of samples. After applying horizontal and vertical flipping in addition to rotation with 15°, the total number of samples increased to 112,920 images. 13% of the images are used for testing while the remaining samples are divided into 75% for training and 25% for validation. From patient's point of view, the images are divided into 14 patients for training, 4 patients' data for validation, and 2 patients' data for testing (patients no. 5 and no. 20).

### 2.2. The Model

The proposed model extends the main feature of 2D U-Net [16] that concatenates the output of each layer in the contracting path to the inputs of the layer on the same level on the expansion pass to limit the effect of the loss in the high level feature during the convolution and pooling process. The model consists of two stacked U-Net with total 4 paths, B1 and B2 are the contracting and expansion path of the first U-Net while B3 and B4 are the components of the second U-Net as in Figure 1. Each U-Net consists of 4 levels at each path in addition to one level to connect the contracting and expansion paths. The number of filters at the contracting path starts with 64 and is increased by 200% for the next level until it reaches 1024 filter at level 5. As for the expansion path, the number of filters is decreased by 50% as the level goes up, reaching the initial 64 filters at the topmost level. The input image size is of 256 × 256 pixels and is decreased by 50% after each level on the contracting path due to the maxpooling process to reach the minimum image size with 16 × 16 at level 5, then start to increase by 50% with each level of upsampling on the expansion path. The output feature maps have equal size at each level on both U-Net paths as shown in Figure 2.

Each path consists of a series of layers to construct a block at each level. The blocks on B1 follow the typical architecture of a convolutional network. It consists of two convolutional layers with filter size 3 × 3 (unpadded convolutions), each followed by an exponential ReLU (ELU) or rectified linear unit (ReLU) at levels 4 and 5, a 2 × 2 max pooling operation with stride 2 for downsampling, and ends with dropout layer with 50% rate. After each block, the number of feature channels will be doubled. The maxpooling and dropout layers are excluded from the block at level 4. The blocks in the expansion path (B2) consists of an upsampling of the feature map followed by a 2 × 2 convolution (upconvolution) that halves the number of feature channels, a concatenation with the corresponding feature map from the contracting path, and two 3 × 3 convolutions, each followed by an ELU or ReLU and a dropout with 45% rate. The blocks in B3 are similar to B1 except that the former starts with a concatenation of the feature map from the corresponding expansion path in B2 with the feature maps from the previous level in the contracting path in B3, then followed by similar layers as in the blocks on B1 (i.e., Conv, Conv, maxpooling, and dropout). The building blocks on B4 have the same structure as B2 except that it concatenates 4 feature maps before applying the sequence of (Conv, Conv, and Dropout). The first feature map that comes from the previous upsampled level in B4 will be concatenated with the feature maps at the corresponding levels from B1, B2, and B3. At the final layer, a 1 × 1 convolution is used to map each 64-component feature vector to the 256 × 256 image mask as shown in Figure 3.

### 2.3. Skip Connections

A model with 2 bridged U-Nets for prostate segmentation [17] introduced a bridge to add the output features from each level at the contracting path of the first U-Net to the inputs of the expansion path of the second U-Net at the same level (blue lines). Our modified model introduces two new bridging connections. One bridge concatenates the output of the expansion path of the first U-Net (B2) to the inputs of the contracting path of the second U-Net (brown lines). The second bridge concatenates the output of B2 to the inputs of B4 (red lines). The final model proposed in this research is a compound model that contains all type of bridging connections. The novel architecture has used all the previously generated feature maps from all paths of the two U-Nets and concatenated them to the inputs of the last expansion path. We hypothesize that by concatenating all previously generated feature maps, the proposed model can decrease the loss of both high-level and low-level features (see Figure 3).

### 2.4. Feature Concatenation

There are two types of operations to combine the features through the bridge and skip connections. Addition operator applies a pixel-wise summation operation and generates one layer for all the input layers. Concatenation operator stacks all the feature maps together along the feature map dimension with depth equal to the number of input layers. We used concatenation with all skip connections and bridge connections since concatenation operation increases the features space by combining the high-level and low-level features. Therefore, the subsequent convolutional operation is able to learn new features that are dependent on both high-level as well as low-level features (see Figure 4).

In comparison, we created another version of the model started with 32 filters applied on the first layer then increased by 200% on the next level to reach 512 filters applied at the deepest level.

### 2.5. Objective and Loss Function

In fact, the U-net, an end-to-end segmentation network, is a classification of each pixel. Most of the deep learning networks use the cross-entropy as a loss function for pixel-wise classification to segment an image into different regions. However, the samples in the dataset we use are only for liver area, and the ratio of positive and negative samples is about 1 : 15, an extremely uneven distribution. If crossentropy function is used in our training process, the result will be biased towards the negative samples.

In view of the above, we implement the Dice loss, a loss function based on Dice similarity coefficient (DSC). The Dice similarity coefficient is a statistical metric that measures the similarity between two sets of data. It has become one of the broadly used metrics in the validation of image algorithms as in

(1) $$\begin{array}{c} \text{Dice}=\frac{2*\;|\;X\cap Y\;|\;}{\left|X\;\right|+\;|\;Y\;|\;}, \end{array}$$

where *X* and *Y* are two sets of pixels of ground truth (masks) and the predicted liver, respectively. ∣*X*∣ is the number of elements in set *X*. ∩ represents the set intersection. The loss function *L*_Dice_ is the difference between the ground truth and the predicted mask as in

(2) $$\begin{array}{c} L_{\text{Dice}}=1-\text{Dice}. \end{array}$$

### 2.6. Training and Testing

The testing samples represent 13% (14,560 images) of the total samples of 3Dircadb1, whilst the remaining samples are divided into training and validation with percentage 75% (74,680) and 25% (14,560). All models trained for 10 epochs with learning rate 1*e*^−5^ using Adam optimizer [38]. All training and testing images were scaled from 512 × 512 to 256 × 256 due to the limitation of computing resources. Training parameters are shown in Table 1.

During the testing phase, each model was evaluated with two groups of data. Firstly, the models were tested using the original testing data without applying any augmentation technique (normal data). Secondly, the models were evaluated using the data after augmentation including all vertically and horizontally flipped images in addition to all 15° step rotated images (augmented data). The results are shown in Tables 2 and 3, respectively.

### 2.7. Hardware and Software

For training and testing, we used Intel® Core™ i7-6700 CPU @ 3.40 GHz×8, with 16 GB RAM and GPU GeForce GTX 1080/PCIe/SSE2 with 8 GB RAM. Our model was implemented using python 2.7.3, for Keras 2.1.1, with TensorFlow 1.2.1, Theano 0.8 for Ubuntu 14.04.05.

## 3. Results and Discussion

We refer to the model by the number of filters at the deepest level. For example, (compound-512) which represents the compound model with filters starts with 32 and ends with 512 at the deepest level, whilst (compound1024) which represents the compound model with filters starts with 64 and ends with 1024 at the deepest level. To compare our results with the original U-Net [16] and 2-Bridged U-Net [17], we conducted two groups of experiments based on the filter structure of the base U-Net. The first group used base U-Net with (32-➔512) while the second group used base U-Net with (64➔1024).

The evaluation metrics of the medical image segmentation algorithms include but not limited to Intersection over Union (IOU) or Jaccard index, Dice similarity coefficient (DSC or Dice), precision, and recall. We use Dice to evaluate and compare our approach with other related work because it is the common metric for most of liver segmentation methods [10, 19, 20, 24, 28–30, 32–36].

The results in Table 2 highlight the key findings. The model U-Net-1024 recorded higher accuracy than U-Net-512. The models based on the modified connections and compound connections recorded higher accuracy than the original connections with both structures 32-512 and 64-1024. The models compound-512 and compound-1024 recorded the best accuracy over original and modified connections for both filter structures 32-512 and 64-1024, except that the modified model with 64-1024 recorded higher accuracy than that of the models with 64-1024 filters when testing with augmented data. Using the filter structure 64-1024 recorded higher accuracy over the filter structure 32-512 except for compound connections. The best overall accuracy for testing with and without augmented data were recorded for compound model using 32-512 filters structure as shown in Figure 5.

The findings came in line with the main hypotheses that by adding the high level feature-maps from the contraction path of the U-Net to the feature-maps on the same level of the expansion path will reduce the loss of the feature that may be caused due to the convolution and pooling operations. The modified model and the compound models add extra bridging connections from the first U-Net to the final expansion path of the second U-Net and have shown better performance over the original model. Although the original 2-bridged U-Net used filters structure 32-512, the results show that using filter structure of 64-1024 recorded higher accuracy because the number of training parameters is higher than the parameters of the model with filters 32-512 for both original and modified models where only one skip connection had been used to transfer the feature maps from the first U-Net to the second U-Net. The compound model has demonstrated that using two skip connections to transfer the feature maps to the second U-Net doubles the size of feature space at the second U-Net, enhances the model performance, and decreases the need of increasing the number of filters to 64-1024 (Figure 5). On the other hand, when the size of the feature space at the second U-Net is doubled due to the compound connections, the number of learnable parameters would also be doubled for all the deconvolutional layers in the second U-Net. It has more significant impact on the filter structure of 64-1024 than that of 32-512. That is, the compound model with the filter structure of 64-1024 is more likely to overfit than the compound model with the filter structure of 32-512. This could explain as to why the compound model with the filter structure of 32-512 had better testing performance in terms of the Dice coefficient than the compound model with the filter structure of 64-1024.

The sample results in Figure 6 illustrated that using 64-1024 filters with all models decreased the over segmentation because the number of the high-level and low-level features on the contracting path increased by 200% that will allow the models to learn more global features. In case of the modified and compound, adding the extra skip connections that concatenate all the previously generated features to the final expansion path reduced the false positive and over segmentation artefacts. Although a few images are segmented with better accuracy using the modified model with 64-1024 filters (h column), the compound model in general recorded the best accuracy with both filters' structure.

Column b shows the results of liver segmentation using the original structure of U-Net with 32-512 filters. The results suffer from artefacts near the boundaries of the liver because the loss in the global features during the downsampling propagated to the following convolutional layers of the next deeper levels. Similar loss happened due to the fusion of the features on the expansion path which indicates that the skip connections in the original U-Net is not enough to overcome the features loss. The segmentation using the original structure of the 2 Bridged U-Net enhanced the accuracy for the images where the liver size is relatively smaller in rows 1 and 2 at column c. On the other hand, the output for the images where the liver size is larger have suffered from oversegmentation because the skip connections from the expansion path at the first U-Net (B2) were concatenated to the contracting path at the second U-Net only, whilst the feature maps from (B1) were transferred directly to (B4) only Figure 1 (original bridge). Column d illustrates the improvement of the output and decreased the oversegmented artefacts because the skip connections of the modified bridge model transferred the low-level features from (B2) directly to be concatenated to the expansion path (B4) at the second U-Net. The compound bridge results in column (e) show the significant enhancement of the performance for all images with small and large liver size because the concatenation of all output feature maps from all the previous paths to the final expansion path of the second U-Net has recovered the loss of the high-level and low-level features. The accumulative residual connections increased the feature space and allowed the model to learn more features by concatenating all the previously generated high-level and low-level feature maps from all the previous paths. Columns (f, g, h, and i) show the results of the models using filter structure 64-1024. Generally, the overall accuracy with 64-1024 models is higher than the models with filter structure 32-515 because of the number of filters, and feature maps generated are increased by 100%. In rare cases, the compound model suffers from undersegmentation at some images with small size liver rows 1 and 2 at column (i) because the number of features transferred from the previous paths to the final path is large and might contain redundant features which increased the false negative for the images with smaller liver size.

The results in Table 3 compared our models with the state-of-the-art approaches that used the same dataset 3Dircadb for liver segmentation. In this paper, we used 14 patients' data for training and 4 patients' data for validation with 80 : 20 ratio and 2 patients' data for testing. In [20], it used 15 patients' data for training and validation and 5 patients for testing; however, it did not specify which patient numbers were used for testing. In [28], 15 patients' data were used for training and testing with 2-fold crossvalidation. In contrast, [32] did not mention any details about the data splitting approach for training, validation, and testing. We used the mean values of the Dice of all the tested images as the accuracy without calculating the STD or tolerance as the way the results were presented in [24, 28].

Christ et al. [28] proposed a cascaded CNN for liver and lesion segmentation with preprocessing the image to convert it to HU values and postprocessing in 2D with a 3D dense conditional random field (CRF) approach. Although their recorded results exceeded the U-Net performance with 94.30%, our compound model outperformed their results with 94.42%. Wang et al. [32] converted the DICOM images to Hounsfield Unit, then used a window of the specific HU for the liver. Replacing the Conv layers at each level with a dense connection blocks significantly increased the number of layers, and the network ended up similar to 5 dense blocks; each block contains 5 U-Nets of 2 levels. Their model is very complicated and computationally expensive with very large number of layers and connections. It is not clear if the stated results were based on testing with 3Dircadb dataset or LiTS as the model was tested on both datasets. It is evident that our compound model outperformed all the benchmarked models stated in [32]. The performance of the proposed compound model is comparable to that of the densely connected U-Net (DC U-Net). Seo et al. [20] included the residual path and a design of object-dependent upsampling to U-Net structure. The network tried to avoid duplication of low-resolution information by adding block or residual layers on the skip connection while it used only one U-Net.

The original architecture of the U-Net model [16] was reimplemented for comparison purpose in this paper as it was the case in [28, 32]. Note that Wang et al. [32] applied preprocessing technique to convert the Dicom images into Hounsfield Unit (HU) to prevent the loss of information when the whole image pixel values are scaled into the range 0-255. Specifically, the raw CT slices are windowed to a Hounsfield Unit range of -100 to 400 HU to neglect organs and tissues that are not of interest. Christ et al. [28] followed the same preprocessing technique and additionally applied histogram equalization for contrast enhancement followed by augmenting the images to increase the number of samples using translation, rotation, and adding Gaussian noise. On the contrary, we did not use any preprocessing techniques but directly converted the Dicom images to pixel values within the range 0-255. Furthermore, whilst [28] used 15 out of 20 patients' data for training, validation, and testing with 2-fold crossvalidation, we used 14 patients' data for training, 4 patients' data for validation, and 2 patients' data for testing. Our testing data might be not included in the 15 patients' data used in [28]. On the other hand, Wang et al. [32] did not mention the methods that used for data splitting. Hence, it explains the discrepancy between the results of our implementation of the U-Net and the results presented in [24, 28].

Our training and testing data were rescaled to 256 × 256 which is 50% of the size of the original images. While [20] used the original image size 512 × 512, [28] and [32] did not mention if they used the original data size or rescaled it. Although scaling the images to smaller size might cause the loss of some features, our proposed models outperformed most of the other models in terms of Dice coefficient (see Table 3). We also plan to work with original image size 512 × 512 in the future for potentially more accurate liver segmentation.

Our approach did not apply any preprocessing technique to the images but directly normalized the DICOM images' pixel intensity to the range 0-255. It thus produced different pixel intensity mapping for the liver region because 3Dircadb1 database contains DICOM image with various HU range. Effectively, the variations of the pixel intensity for the liver region act as an image augmentation technique. Note that image augmentation techniques, such as adding noises to image intensity values amongst others, have been shown to be very useful for deep learning based models. We have compared our results with methods that applied image calibration or windowing process based on Hounsfield Units [28, 32]. Our results are comparable or better in terms of the Dice coefficient. We plan to add preprocessing step that includes windowing process in our future work to compare its effectiveness with the models that do not apply the windowing process.

Although 3D CNNs can process volumetric information, they have some disadvantages. Due to the increased dimension, 3D CNNs require higher computational cost. Besides, the large number of parameters may result in higher risk of overfitting, especially when encountering small datasets. Moreover, the GPU requirement of 3D CNNs is impractically expensive, which hinders their further clinical application. Our model is implemented based on 2D U-Net architecture where each CT slice is treated as input image that is independent of other slices. The proposed model has much lighter computational cost but higher inference speed. In our future work, the information between adjacent slices could be taken into consideration.

## 4. Conclusions

In this paper, we proposed a novel segmentation method, and the experimental results show that stacking two U-Nets and adding three bridging connections from the first U-Net to the second U-Net can significantly improve the accuracy of liver segmentation. The accumulative approach of concatenating the feature maps from the previous layer with all the previously generated features at the same level from all the previous paths of the 2 stacked U-Nets significantly reduced the loss of global features and low level features during the pooling and upsampling and outperformed most of the recent approaches. The model results are robust against noise as it did not use any preprocessing or postprocessing. Our model used augmentation techniques to overcome the shortage of the medical data with manually annotated masks, and it showed a significant improvement in the performance when testing with the augmented data.

## Figures and Tables

**Figure 1:** The architecture overview of the proposed 2 stacked U-Net main structure. B1 and B2 are contracting and expansion path for the first U-Net while B3 and B4 are the contracting and expansion path of the second U-Net. The colored lines represent the bridging connections between the different paths. Original, modified, and compound are three different structures of the bridging connections.

**Figure 2:** The proposed compound W-Net model structure. The model connects two U-Nets with 3 bridging connections (blue, red, and brown) and one skip connection in each U-Net (dark blue).

**Figure 3:** Detailed architecture of the model with the layers in each block for all branches B1, B2, B3, and B4.

**Figure 4:** The difference between concatenation and addition operations.

**Figure 5:** The accuracies in percentage for trading, validation, and testing using normal data and testing using augmented data for all models' structure (U-Net, original bridge, modified bridge, and compound bridge) with both filter structures (32 ➔ 512) and (64➔ 1024).

**Figure 6:** Comparison of testing results. (a) Ground truth, (b) U-Net, (c) bridged 2U-Net, (d) our modified stacked U-Net, (e) our compound 2U-Net. All (b–e) with filter structure 32-512. All (f–i) with filter structure 64-1024.

**Table 1:** Model parameters for training.

Parameters	Values
Image size	256 × 256
Number of epochs	10
Learning rate	1*e*^−5^
Filter size	3 × 3
Pooling size	2 × 2
Dropout rate contracting path	0.5
Dropout rate expanding path	0.4
Filters per layer	Previous layer′s filters × 2

**Table 2:** The accuracies of training, validation, testing using normal images, and testing using augmented images for all four types of models (U-Net, original, modified, and compound) using both versions with (32➔ 512) and (64➔ 1024) filters structure. The accuracy represents the value of Dice similarity coefficient.

Model	Filters	Training	Validation	Testing	
		Dice	Dice	Normal data Dice	Augmented data Dice
U-Net [16]	32-512	0.9650	**0.9800**	0.4649	0.6007
Bridge U-Net [17]	32-512	0.9755	0.7065	0.7321	0.6031
Our modified bridge	32-512	*0.9785*	0.6702	0.7912	0.6010
Our compound model	32-512	0.9752	0.9011	**0.8988**	**0.9442**
U-Net [16]	64-1024	0.9740	0.9150	0.5873	0.7593
Bridge U-Net [17]	64-1024	0.9738	0.8775	0.7989	0.7534
Our modified bridge	64-1024	*0.9812*	*0.9250*	0.8137	*0.8368*
Our compound model	64-1024	**0.9812**	0.9113	*0.8303*	0.7836

**Table 3:** Quantitative comparison between our models and other models using 3Dircadb dataset.

Model	Dice	Testing	
	%	Normal data Dice %	Augmented data Dice %
U-Net [16]		46.49	60.07
Bridge U-Net [17]		73.21	60.31
Our modified bridge		79.12	60.10
Our compound model		**89.88**	**94.42**
U-Net [32]	92.6 ± 2.2		
FCN-8 s [32]	92.1 ± 1.5		
3D DSN [32]	92.8 ± 1.4		
DecNet [32]	90.1 ± 1.0		
FCN [32]	93.30		
Cascaded UNet+CRF [32]	93.10		
DC U-Net [32]	94.9 ± 2.0		
mU-Net [20]	96.01 ± 1.8		
UNET [28]	72.90		
Cascaded UNET [28]	93.10		
Cascaded UNET +3D CRF [28]	**94.30**		

## Data Availability

The dataset 3Dircadb1 for liver CT scans and the associated masks for each liver are publicly available on [37] in DICOM format.
